This article has been retracted.

# Rapid and sustained antidepressant effects of intravenous ketamine in treatment-resistant major depressive disorder and suicidal ideation: a randomized clinical trial

**DOI:** 10.1186/s12888-024-05716-0

**Published:** 2024-05-07

**Authors:** Ahmad Zolghadriha, Afagh Anjomshoaa, Mohammad Reza Jamshidi, Farnaz Taherkhani

**Affiliations:** 1 Department of Psychiatry, Shahid Beheshti Hospital, Zanjan University of Medical Sciences, Zanjan, Iran; 2 Zanjan Metabolic Diseases Research Center, Zanjan University of Medical Sciences, Zanjan, Iran; 3 Department of Anesthesia, School of Medicine, Mousavi Hospital, Zanjan University of Medical Sciences, Iran Zanjan,

**Keywords:** Ketamine, Major depressive disorder, Suicide ideation, Clinical trial

## Abstract

**Background:**

Major depressive disorder (MDD) is the most disabling and burdensome mental disorder, negatively affecting an individual’s quality of life and daily functioning. the current study was conducted with the aim of investigating the clinical effects of intravenous ketamine on symptoms of MDD and suicidal ideation.

**Methods:**

The current randomized clinical trial was carried out on 64 patients diagnosed with treatment-resistant major depressive disorder between April and August 2022. The participants were randomly assigned to two groups: the intervention group received a dose of 0.5 mg/kg of ketamine, while the control group received normal saline. The Montgomery-Asberg Depression Scale and Beck’s Suicidal Ideation Scale were utilized to assess depression and suicidal ideation, respectively.

**Results:**

One hour after the administration of ketamine treatment, there was a notable and significant improvement in both depression symptoms (35.16 ± 8.13 vs. 14.90 ± 10.09) and suicidal ideation (6.74 ± 6.67 vs. 0.42 ± 1.52). Moreover, there were statistically significant differences in depression scores between the two groups at one hour, four hours, one day, three days, one week, one month, and two months after the administration of ketamine (p-value < 0.001). However, ketamine recipients frequently experienced side effects such as increased heart rate, headache, dizziness, and dissociative syndrome symptoms.

**Conclusion:**

The observed rapid onset of action and sustained effect demonstrate the potential of ketamine to provide relief from depressive symptoms in a shorter timeframe compared to traditional treatment approaches. These findings contribute to the growing body of evidence supporting the use of ketamine as a valuable therapeutic option for patients with treatment-resistant depression.

**IRCT registration:**

IRCT registration number: IRCT20210806052096N1; IRCT URL: https://www.irct.ir/trial/62243; Ethical code: IR.ZUMS.REC.1400.150; Registration date: 2022-04-09.

## Introduction

Major depressive disorder (MDD) is the most disabling and burdensome mental disorder, negatively affecting an individual’s quality of life and daily functioning [1]. Globally, according to the World Health Organization (WHO), more than 264 million people of all ages suffer from depression, and the lifetime prevalence of MDD ranges from 2 to 21% [2]. MDD is attributed to over eight hundred thousand deaths by suicide [3]. The economic burden of MDD in the United States was approximately $210.5 billion annually, encompassing direct healthcare costs, productivity losses, disability, and the impact on caregivers [4].

Despite the significant impact of MDD on various aspects of individuals’ lives, including emotional well-being, physical health, cognitive functioning, work performance, and the increased risk of other health issues, there is no effective and safe medications, so up to one-third of individuals are considered to be treatment-resistant [5, 6]. Furthermore, there is often a delay of more than two weeks in the onset of clinical effects for many medications, during which the patient’s symptoms may worsen, and in some cases, even suicidal ideation may occur [7, 8]. Suicidal ideation in MDD patients is considered a critical emergency and requires prompt attention and immediate treatment due to the severity of the condition [7].

Ketamine, known for its rapid response, has shown promising results as a medication in the treatment of major depressive disorder (MDD), especially in cases where other treatments have proven ineffective. It acts as an antagonist of the N-methyl-D-aspartate (NMDA) receptor, blocking the activity of glutamate, an excitatory neurotransmitter. This modulation of glutamate levels may contribute to the restoration of neurotransmitter balance in the brain, potentially leading to an improvement in mood [9, 10]. Moreover, Ketamine has been observed to enhance the production of brain-derived neurotrophic factor (BDNF), a protein crucial for promoting the growth and survival of neurons. This augmented neuroplasticity potential may contribute to the repair or strengthening of damaged neural circuits associated with depression [10, 11].

Recent randomized controlled trials have yielded compelling evidence supporting the therapeutic efficacy of ketamine treatment in MDD [12–15]. However, there are some concerns regarding the potential side effects of ketamine, including tolerability, dissociation, vasomotor symptoms, headache, nausea, vomiting, urinary incontinence, as well as short-term and long-term safety [16].

Considering the diverse approaches used in terms of appropriate dosage, administration, and route of ketamine, when utilized as an antidepressant medication, it is necessary to conduct further studies to thoroughly investigate the clinical efficacy and potential side effects of this medication. Therefore, the current study was conducted with the aim of investigating the clinical effects of intravenous ketamine on symptoms of MDD and suicidal ideation.

## Material & method

### Study design and setting

To assess the effects of intravenous ketamine on major depressive disorder and suicidal ideation, we conducted a 2-month, randomized, controlled, assessor-blinded clinical trial. This study was conducted on 64 patients with treatment-resistant major depressive disorder in Shahid Beheshti Hospital, Zanjan, Iran, from April and August 2022.

### Ethical considerations

The research protocol received approval from the research ethics committee of Zanjan University of Medical Sciences (code: IR.ZUMS.REC.1400.150). Additionally, this study was registered with the Iranian Registry of Clinical Trials (code: IRCT20210806052096N1). After explaining the purpose of the study, verbal and written consent was obtained from all participants. They were also reassured that their participation was voluntary and that their personal information would remain confidential.

### Participant selection, and sampling

The study participants were recruited from outpatients referred to the psychiatric clinic at Shahid Beheshti Hospital and private offices. Two experienced psychiatrists from the Department of Psychiatry at Zanjan University of Medical Sciences independently conducted structured interviews to diagnose Major Depressive Disorder (MDD) in accordance with the Diagnostic and Statistical Manual of Mental Disorders, Fifth Edition (DSM-5) criteria.The inclusion criteria were as follows (1) age between 25 and 60 years; (2) Diagnosis of major depressive disorder based on DSM-5 criteria, (3) lack of significant improvement in depressive symptoms despite adequate trials of at least two different antidepressant medications; 3) not pregnant, or breastfeeding; (4) Absence of contraindications for ketamine treatment such as uncontrolled hypertension, active substance abuse, or a history of psychosis. (5) competent to provide informed consent; (6) Montgomery-Asberg Depression Scale score above 25.

Exclusion criteria included allergy or hypersensitivity to ketamine, unwillingness to continue participating in the study, worsening patients’ general condition.

The process of participant selection has been described in the Fig. 1. The eligible patients who met the inclusion criteria were included in the study using the convenience sampling method.

**Fig. 1:** The trend of depression score in trial (ketamin), and control (placebo) groups

The sample size was determined through the utilization of GPower 3.1 software, based on a preliminary experiment effect size (d) of 0.50. The power analysis revealed that 58 participants would achieve 80% statistical power with a two-sided α of 0.05 and an effect size (d) of 0.50. Taking into account a 10% dropout rate, the intended total sample size was established at 64 participants.

### Randomization, allocation concealment, and blinding

The patients were randomly assigned to two groups using block randomization, with each block consisting of four participants. The intervention (A) and control (B) groups were determined by permutation blocks of four, with two participants assigned to the ketamine treatment group and two participants assigned to the placebo group. The status of four patients was determined for each block using a table of random numbers, ensuring a balanced distribution of samples across both groups.

To ensure the concealment of random allocation, sequentially numbered and sealed opaque envelopes of the same shape were utilized, and neither the researcher’s nor the participants’ opinions had any impact on the assignment of individuals to the intervention or control group. Furthermore, to minimize selection bias, the allocation of participants to either the trial or control group was carried out by a researcher who was not involved in data collection. whereas participants in the control group were prescribed normal saline; both psychiatrist and patients were kept blind to the type of drug being administered.

### Interventions

Participants in the trial group were administered a prescription of 0.5 mg/kg intravenous ketamine (Ampule KETAMIN ROTEXMEDICA Injection 50 mg/ml, 10 ml, Nature Made Germany), The drug injection was administered by a psychiatrist, and patients from both groups were instructed to continue taking their anti-depressant medications. Heart rate, blood pressure, and blood oxygen saturation were monitored at regular intervals during the infusion, as well as at 60 and 120 minutes’ post-infusion.

The severity of depression was assessed using the Montgomery-Asberg scale immediately prior to the injection, at 60 min, 120 min, and 240 min after the start of the injection, as well as at 1 day, 3 days, 7 days, one month, and two months’ post-injection.

### Outcomes measurement

The Montgomery-Asberg Depression Rating Scale (MADRS) is a widely used clinician-administered rating scale designed to assess the severity of depressive symptoms in individuals with major depressive disorder. This consists of 10 items that cover various symptom domains of depression, including mood, feelings of sadness, tension, sleep disturbances, appetite changes, concentration difficulties, lassitude, pessimism, suicidal thoughts, and inner tension. Each item is rated on a scale of 0 to 6, with higher scores indicating greater severity of symptoms. The total score ranges from 0 to 60, with higher scores indicating a greater overall level of depression. This scale has good validity, and reliability in Iranian population [17].

Beck’s Suicidal Ideation Scale (BSIS) was used as a self-report questionnaire specifically designed to assess the presence and severity of suicidal thoughts in individuals. The BSIS consists of 19 items that measure various aspects of suicidal ideation, including intensity, frequency, and specificity. Each item is scored on a 3-point Likert scale, ranging from 0 to 2, with higher scores indicating a higher level of suicidal ideation. The total score on the BSIS can range from 0 to 38, with higher scores indicating a greater severity of suicidal ideation. The scale also includes three subscales: the wish to die, the active suicidal desire, and the passive suicidal desire subscales. The validity, and reliability of this questionnaire was approved among Iranian population [18].

### Statistical analysis

Data analysis was conducted using SPSS software version 24. Descriptive statistics were employed to present the sociodemographic and clinical variables. T-tests, Mann-Whitney U test, chi-square test, and repeated measures analysis of variance were performed using a forward selection procedure with a significance level of 0.05 to assess the comparison of depression and suicide scores between two groups (experimental and control) at multiple time points (before, 1 h, 4 h, 1 day, 3 days, 1 week, 1 month, and 2 months after the investigation).

## Results

The mean age of participants in the ketamine and placebo groups was 38.77 ± 9.13 and 40.06 ± 7.65 years, respectively, with no statistical difference observed. Additionally, there were no statistical differences between the two groups in terms of gender, education, marital status, residency, lifetime suicide attempts, age at onset of MDD, duration of depression treatment, duration of current episode, and lifetime number of MDD (p-value > 0.05) (Table 1).

**Table 1:** Demographic, and clinical characteristic of participants with major depressive disorder

Variables	Trials (*N* = 32) Number (percent)	Controls (*N* = 32) Number (percent)	*p*-value
Age	38.77 ± 9.13	40.06 ± 7.65	0.55
Gender			
Women	14(43.75)	12(37.50)	0.46
Men	14(43.75)	12(37.50)	
Education			
University	20(62.5)	17(53.12)	0.29
Non-university	12 (37.50)	15 (46.87)	
Marital status			
Married	24(75)	21(65.62)	0.26
Single	8 (24)	11(34.37)	
Residency			
Rural	11(34.27)	9(28.12)	0.43
Urban	21(65.62)	23(71.87)	
Number of life-time suicide attempt			
0	20(62.50)	24(75)	0.07
1–3 times	9(28.12)	7(21.87)	
> 3 times	3(9.37)	1(3.12)	
Age at onset of MDD^*^	27.51 ± 10.02	29.74 ± 5.45	0.27
Duration of depression treatment ^*^	11.64 ± 3.65	10.29 ± 2.16	0.08
Duration of current episode (week) ^*^	12.49 ± 2.93	13.62 ± 3.02	0.13
Number of previous episodes of MDD^*^	5.36 ± 1.31	6.02 ± 1.70	0.09

*data was reported as Mean ± SD, MMD: Major depressive disorder

Before the intervention, there were no statistically significant differences in the mean scores of depression between the two groups (p-value = 0.14). However, one hour after the treatment, there was a rapid improvement in the symptoms of depression, as evidenced by the lower scores observed (35.16 ± 8.13 vs. 14.90 ± 10.09), and this relationship was statistically significant (p-value < 0.001) (Fig. 2). Furthermore, there were statistically significant differences in depression scores between the two groups at four hours, one day, three days, one week, one month, and two months after ketamine treatment (p-value < 0.001) (Table 2).

**Fig. 2:** The trend of depression score in trial (ketamin), and control (placebo) groups

**Table 2:** Response rates in depression symptoms in patients with major depressive disorder following intravenous ketamine or placebo

Depression score	Trial	Control	*p*-value
Before intervention	35.16 ± 8.13	32.51 ± 5.66	0.14
One hours	14.90 ± 10.09	29.77 ± 4.56	< 0.001
Four hours	9.83 ± 11.13	28.03 ± 3.74	< 0.001
One day	11.16 ± 11.75	28.61 ± 3.87	< 0.001
Three day	10.41 ± 13.89	28.67 ± 3.53	< 0.001
One week	11.32 ± 13.43	29.38 ± 4.42	< 0.001
One month	15.38 ± 13.27	29.48 ± 4.21	< 0.001
Two month	17.09 ± 13.45	28.70 ± 3.58	< 0.001

Assuming variable normality, a repeated measure analysis of variance was conducted to examine the effect of intravenous ketamine on depression symptoms at multiple time points during the follow-up period. However, the assumption of covariance matrix uniformity was not met (P-value < 0.001). Since the amount of Greenhouse–Geisser epsilon-corrected value was approximately 0.62 for depression, the corrected value was used to adjust the results accordingly. Considering the significant intragroup effect and the presence of more than two groups, the Bonferroni post hoc test was utilized. The results of this test indicated that all pairwise comparisons before and after the intervention yielded statistically significant differences (*P* < 0.001). This suggests that the intervention had a significant impact on depression symptoms at all assessed time points (Fig. 1).

Vital signs and oxygen saturation were monitored up to two hours after treatment and compared between the two groups. There was no significant difference between the two groups in terms of oxygen saturation, systolic blood pressure, and diastolic blood pressure (p-value > 0.05). The only significant difference observed was in the heart rate, which was higher in the group receiving ketamine (*p* = 0.001) (Table 3).

**Table 3:** Assessment of blood pressure, heart rate, and blood oxygen saturation, immediately, one hour, and two hours after ketamine and placebo administration

	Time	Trials	Controls	*p*-value
Heart rate	Immediately	98.70 ± 15.02	78.70 ± 6.44	0.001
	One hour	82.33 ± 12.01	78.25 ± 6.30	
	Two hours	80.10 ± 8.93	78.37 ± 6.25	
O2 saturation	Immediately	96.96 ± 1.79	96.74 ± 1.48	0.49
	One hour	97.26 ± 1.38	96.73 ± 1.25	
	Two hours	97.36 ± 1.29	96.77 ± 1.36	
Systolic blood pressure	Immediately	115.06 ± 20.44	113.33 ± 22.74	0.05
	One hour	108.90 ± 27.15	116.66 ± 10.09	
	Two hours	116.00 ± 4.98	104.96 ± 34.79	
Diastolic blood pressure	Immediately	73.87 ± 6.01	72.96 ± 8.11	0.41
	One hour	75.50 ± 4.30	72.40 ± 7.88	
	Two hours	75.48 ± 4.27	72.41 ± 8.13	

Before the intervention, there was no significant difference in terms of suicidal ideation between the two groups. However, after the intervention, a notable decrease in suicidal ideation was observed specifically in the group that received ketamine treatment (p-value < 0.001) (Table 4).

**Table 4:** Comparison of suicidal ideation score before, and after treatment

	Trial	Controls	*p*-value
Before intervention	6.74 ± 6.67	3.58 ± 2.57	0.11
After intervention	0.42 ± 1.52	3.35 ± 2.80	< 0.001

In the term of side effects, 100% of individuals reported headache and dissocuative syndrome. Additionally, dizziness, nausea, anxiety, and visual disturbances were observed in 56%, 25%, 12.5%, and 6.25% of patients treated with ketamine, respectively (Table 5).

**Table 5:** comparison of side effects between two groups

	Ketamine group	Placebo	*p*-value
anxiety	4 (12.5)	0	0.11
Headache	32 (100)	0	0.24
dizziness	18 (56.25)	0	0 < 001
nausea	8 [24]	0	0.005
Syncope	0	0	1.0
visual illusion	2 (6.25)	0	0.49
Dissocuative syndrome	32 (100)	0	0 < 001

## Discussion

The results of the present study highlight that a single intravenous dose of 0.5 mg/kg of ketamine had a rapid, and significant antidepressant response in patients with MDD who had previously not responded to at least two antidepressant trials. Within one hour of treatment, a noticeable improvement in the patient’s clinical symptoms occurred, and this improvement continued for up to two months after the intervention. Despite clinical improvement, an increase in heart rate, headache, dizziness, and dissocuative syndrome symptoms were frequently observed in ketamine recipients.

The initial evidence of the clinically rapid antidepressant effects of ketamine was documented in a study conducted by Berman et al. in 2000, that they reported individuals with treatment-resistant depression exhibited a notable improvement in their depressive symptoms within hours after receiving a single intravenous dose of ketamine [19]. Another retrospective study on 213 MDD patients found that the infusion of 0.5 mg/kg of intravenous ketamine in four doses over a period of 7–14 days resulted in a response rate of 27% and a remission rate of 13%. Furthermore, patients who received intravenous ketamine reported experiencing anxiolytic effects, improvements in overall psychosocial function, and a reduction in suicidal ideation. Similar to our study, common side effects observed after ketamine treatment included anxiety, headache, derealization, depersonalization, confusion, dizziness, nausea, drowsiness, double vision, blurred vision, and an increase in systolic and diastolic blood pressure. It is important to note that their study lacked a control group and follow-up assessment [15].

The rapid onset of action and sustained improvement for several days to two months after treatment make ketamine a potential option for individuals with treatment-resistant depression.

Previouse researches followed the efficacy of ketamine for less than two weeks. The results of one meta-analysis on 10 studies with 368 subjects indicated that the administration of 0.5 mg/kg ketamine had therapeutic effects on depressive symptoms at 24 and 72 h, as well as on day 7 after treatment [20]. Another RCT demonstrated that repeated treatment with low doses of ketamine (0.5 mg/kg, three times) is more effective than ECT and can induce rapid antidepressant effects in patients with MDD, and its antidepressant effects persisted for up to one week after the last injection [21].

Our finding suggests that a single dose of ketamine can rapidly reduce suicidal ideations in individuals with treatment-resistant depression. Research studies have demonstrated that ketamine, particularly in the form of intravenous infusion, can rapidly and significantly reduce suicidal thoughts in individuals with MDD who are at high risk for suicide [7, 15]. The anti-suicidal effects of ketamine have been observed to occur within hours or even minutes after administration, making it a potentially life-saving intervention for those in acute distress. These effects have been reported to persist for days or even weeks in some cases [7, 15].

Ketamine is proposed to alleviate several common symptoms of Major Depressive Disorder (MDD), including depressed mood, feelings of guilt or worthlessness, loss of interest in activities, fatigue, changes in appetite, sleep disturbances, and difficulty concentrating [22].

Ketamine’s rapid antidepressant and anti-suicidal effects are believed to be linked to its ability to enhance synaptic plasticity. By blocking NMDA receptors and increasing glutamate release, ketamine activates AMPA receptors, leading to a series of molecular events that promote the growth and strengthening of synapses. This mechanism may help reverse the synaptic deficits associated with depression and suicidal ideation [22, 23]. Moreover, research studies have demonstrated that ketamine administration can induce alterations in the functional connectivity of the brain, ultimately affecting the overall connectome. When considering single ketamine treatment, it has been observed that a single dose can rapidly and transiently modify functional connectivity patterns in various regions of the brain. The precise mechanisms underlying these changes are still under investigation, but it is believed that ketamine’s effects on glutamate transmission and synaptic plasticity contribute to these alterations [24].

Furthermore, there is compelling evidence suggesting that inflammation may play a role in the development of depression. Ketamine has been discovered to possess anti-inflammatory properties, which may help diminish the inflammatory response in the brain and alleviate symptoms of depression [25].

It is worth noting that while the findings of this study are promising, further research is needed to fully understand the mechanisms underlying the antidepressant effects of ketamine and to determine the long-term safety and efficacy of this treatment approach. Additionally, exploring optimal dosing strategies and identifying potential predictors of treatment response will be crucial in refining the use of ketamine as an antidepressant intervention.

## Conclusion

The observed rapid onset of action and sustained effect demonstrate the potential of ketamine to provide relief from depressive symptoms in a shorter timeframe compared to traditional treatment approaches. These findings contribute to the growing body of evidence supporting the use of ketamine as a valuable therapeutic option for patients with treatment-resistant depression.

## Data Availability

The data sets used and analyzed during the current study are available from the corresponding author upon reasonable request.
